RETRACTED

# Research on Sports Health Care Information System Based on Computer Deep Learning Algorithm

**DOI:** 10.1155/2022/1573562

**Published:** 2022-06-30

**Authors:** Xiaojun Ma, Zhenfeng Zhang

**Affiliations:** ^1^School of Physical Education, South China University of Technology, Guangzhou 510640, Guangdong, China; ^2^Zhengzhou University of Aeronautics, Zhengzhou 450046, Henan, China

## Abstract

There are various problems in diagnosing and treating tumor diseases in significant hospitals. The content includes misjudgement and over-surgery issues. For example, the judgment of pulmonary nodules mainly relies on artificial experience, and most of the artificial experience is too radical. This paper is mainly based on the extensive medical data of significant hospitals, extracts the diagnosis and treatment data and digital images of similar cases from the extensive database, classifies them through the deep learning of the computer, and then proposes the control mechanism and the solution of the doctor's misjudgement and excessive medical treatment. This method mainly relies on the CT and MRI digital images of various types of tumor diseases accumulated in the history of major hospitals. Based on the preliminary judgment of each diagnosis and treatment and the results of surgical and pathological examinations, the accumulation of various types of digital images from the history is used. The features are analysed and extracted, the model is built, and finally, a predictive analysis system for this type of tumor is obtained, which can predict the benign and malignant cases of currently occurring cases and avoid the limitations and instability of artificial experience greatest extent. It is proved by experiments and combined with Spearman to remove redundancy. The redundancy removal method SVM_RFE is used for dimensionality reduction. The method can timely correct the misjudgement of the doctor's experience and effectively reduce the instability of the manual, which provides a solution for solving the contradiction between doctors and patients and improving the scientific of diagnosis and treatment.

## 1. Introduction

Human beings have entered the twenty-first century with the development of science and technology, the vigorous development of biological sciences, the rapid development of biomolecules and human genetics, and breakthroughs in human understanding of diseases. In today's increasingly scarce, especially the mismatch between high-quality medical resources and the people's medical needs, the contradiction between doctors and patients is constantly increasing [1]. In the doctor's diagnosis and treatment processing, due to personal negligence or lack of medical literacy, the patient's condition is delayed.

RETRACTED

The cost of tumor patients is enormous, and the misjudgement of doctors will make this problem worse. For patients with malignant tumors who are misjudged as benign tumors by doctors, it will seriously affect the life cycle of patients. There are many influencing factors of wrong-medical treatment, which are the keys to the long-term impact of wrong-medical treatment. Moreover, China currently does not have a systematic correction policy for excessive medical treatment or wrong-medical treatment, which can only be corrected in the case of quite significant wrong-medical treatment. There is a lack of restraint, review, and accountability mechanisms in the policy. There is a lack of systematic corrective action for both mismedical and over-medical treatment, both in policy and technology.

This paper aims to extract relevant parameters and digital images from patient medical records of tumor diseases to establish a scientific benign and malignant classification model. This article collected medical records of 194 patients with pulmonary nodules. This paper first uses the current mainstream method, radionics, to collect texture features from patient medical records. Then, LASSO regression is used to reduce dimensionality, using logistic regression to build a model, and the ROC curve is used to go back to evaluate the model [2]. Feature selection methods are then derived using statistical methods and computer deep learning algorithms and compared with modeling schemes. Finally, Spearman is used to remove redundancy, SVM_RFE dimensionality reduction, and SVM type classification model. This presents the best conclusion in judging benign and malignant pulmonary nodules.

### 1.1. A Framework Analysis of Mechanisms for Identifying Over- and Wrong-Medical Problems

First of all, this research needs to collect a certain number of medical records of tumor patients from the hospital. Conduct an in-depth investigation of these data to ensure the authenticity and reliability of the data, have an in-depth understanding of the hospital's medical procedures and processes, understand the tumor Misjudgement of disease, and propose an assessment model to manage over surgical treatment. Then, the relevant data types are evaluated, and scientific management and control methods are put forward for the diagnosis and treatment errors and excessive medical treatment standards in the hospital [3]. The framework of the management and control process of tumor disease diagnosis and treatment is shown in Figure 1.

The mechanism and method process of wrong diagnosis and treatment and over-medical problem discovery in medical institutions in tumor patients are shown in Figure 1. The framework takes doctors as the subject of subjective cognition from the diagnosis and treatment process and results in higher participation. Separation in evaluation reduces human interference factors and improves the objectivity of evaluation results [4]. Based on obtaining digital image parameters in a large number of medical data, scientific judgments are made on patients' types of diseases and benign and malignant predictions. When a tumor patient goes to the hospital, the doctor needs to carry out a series of inquiry work to obtain the characteristics of the disease and physiological response and then conduct a series of auxiliary medical examinations on the patient. The type of disease is determined, which includes CT images, MRI images, and other digital images. The discovery mechanism of misdiagnosis and overmedication in Figure 1 adds the relevant data of the patient's medical record to the database as a reliable sample medical record.

RETRACTED

### 1.2. Excessive and Incorrect Medical Problem Classification Model

A benign sample of a particular sports injury and a malignant sample of this type of tumor are given as the overall training sample set *D*={(*x*_1_, *y*_1_), (*x*_2_, *y*_2_), ⋯, (*x*_*m*_, *y*_*m*_)}. Among them, *x*_*i*_ is the various image feature parameters extracted from the image data in the medical record and *y*_*i*_ represents the real benign and malignant tumor grade of the patient corresponding to the medical record. The most basic idea of classification learning is to find a partitioning hyperplane in the sample space based on the training set *D*. At the same time, we separate the diagnosis and treatment samples from different categories. Label the classification target disease as *y*_1_. Other types of diseases *y*_2_, ⋯, *y*_*m*_ are uniformly marked as *y*_0_. The ideal goal is to find a partitioning hyperplane that lies “in the middle” of the *y*_0_ and *y*_1_ classes of training samples. Partitioning the hyperplane in the sample space can be described by the following linear equation:

(1) $$\begin{array}{c} \omega^{T}x+b=0, \end{array}$$

*ω*=(*ω*_1_; *ω*_2_; *ω*_3_; …; *ω*_*d*_) is the average vector. It determines the direction of the hyperplane. *b* is the displacement term. It determines the distance between the hyperplane and the origin. The average vector and the displacement can determine the dividing hyperplane *b*. This paper will denote it as (*ω*, *b*). The distance from any point in the sample space to the hyperplane (*ω*, *b*) can be written as

(2) $$\begin{array}{c} r=\frac{\left|\omega^{T}x+b\right|}{\left\|\omega \right\|}. \end{array}$$

Suppose that the hyperplane (*ω*, *b*) can correctly classify the two classes of training samples *y*_0_ and *y*_1_. (*x*_*i*_, *y*_*i*_) ∈ *D*,  *y*_*i*_. If it belongs to the classification target disease *y*_1_, there is *ω*^*T*^*x*+*b* > 0; if it does not belong to the classification target disease *y*_1_, there is *ω*^*T*^*x*+*b* < 0:

(3) $$\begin{array}{c} \left\{\begin{array}{cc} \omega^{T}x+b\geq +1, & y_{i}=y_{1},\\ \omega^{T}x+b\leq -1, & y_{i}=y_{0}. \end{array}\right. \end{array}$$

The sum of the distances from the two heterogeneous support vectors to the hyperplane is

(4) $$\begin{array}{c} \gamma =\frac{2}{\left\|\omega \right\|}. \end{array}$$

The feature selection algorithm for disease classification is as follows:

(1) This paper obtains the LaGrange operator vector of the SVM regular term. The classifier parameters are expressed as follows:
  (5) $$\begin{array}{c} \alpha =SVM-\text{train}\left(X,y\right). \end{array}$$
(2) Calculate the weight vector of each feature vector, that is, the weight vector of clinical index parameters in the input space to obtain the weight of the complete support vector machine:
  (6) $$\begin{array}{c} \omega =\sum_{k}\alpha_{k}y_{k}X_{k}. \end{array}$$
(3) This paper uses a suitable sorting method to sort the weight vectors in the dataset. This suggests that this metric has the most negligible effect of incorrectly classifying the target disease until only one feature remains in the final dataset.
  (7) $$\begin{array}{c} R_{c}=\left|\omega^{2}-\omega^{-{\left(p\right)}^{2}}\right|, \end{array}$$
  where *ω*^2^ represents the weights of the entire SVM and *ω*^−(*p*)^2^^ represents the weight of the support vector machine after removing the *p* feature.

RETRACTED

## 2. The Similarities and Differences between Spearman's SVM Method and the Traditional Radionics Method

### 2.1. Extraction Process of Training Data

The error diagnosis and treatment of SVM and the modeling method of over-medical problems have been described above. The follow-up problem is obtaining better quality training data [5]. This will ensure the inductive attribute ability of the predictive model. The process is shown in Figure 2.

Figure 2 is the training data model extracted from the collected medical database. Including the excellent medical records accumulated in the history of high-quality hospitals, the correctness of the data in the case database collected in the early stage will be directly related to the reliability of the model prediction. Therefore, it is necessary to test the reliability of the early stage data, combining the experience of medical experts and the equipment first [6]. According to the monitoring rules, the relevant information of patients, pathological information, information about drugs prescribed by doctors, and information about surgery should be screened to some extent. The selected data are randomly selected from the database, and the features are comprehensively extracted.

RETRACTED

### 2.2. Construction of a Disease Prediction Model Based on SVM and Similar Expert Prescriptions

The digital images of pulmonary nodules used in this study are shown in Figure 3. In Figure 3, the visible lesion area in the lung lobe page is small, and the right image is the enlarged image of the left lung nodule and the stereo reconstruction. It is difficult for doctors to judge whether the tumor is benign or malignant based on these imaging features alone. It is easy to lead to a wrong judgment of the nature of the tumor.

The tumor diagnosis and management model studied in this paper is divided into four steps. (a) The digital images of N cases of benign and malignant tumors that have been diagnosed are mainly collected, and the N cases are randomly divided into two groups, *X* cases and Y cases. (b) Recognizing images of all samples and extracting *M* information indicators of GLCM, GLRLM, histogram, and form factor, the relevant matrix can be solved. This paper constructs the relevant model research for classification and annotation and uses Y examples to simulate and verify the model's validity.

### 2.3. Comparison of Spearman's SVM Method Used in This Paper with Mainstream Radionics Methods

The control mechanism of these two methods for the wrong diagnosis and treatment of tumor diseases and excessive medical treatment is to obtain digital image parameters from the database and then feedback on the results. The difference lies in the dimensionality reduction of the sample data and linear regression for the classifier Radiomics. It adopts LASSO regression in engineering. SPSS software was used for modeling and analysis to draw relevant conclusions.

### 2.4. Experimental Verification and Results

This paper used the digital image data of 194 pulmonary nodules obtained from the hospital as samples. The test results were quantified by comparing the sampling method of this test with the traditional mainstream methods [7]. The test results verified the effectiveness of the tumor diagnosis and treatment control mechanism proposed in this paper.

### 2.5. Experimental Data Division and Preprocessing

There are 194 cases in the total sample, and 139 cases are diagnosed as benign. This paper analyses the samples of 64 cases. One hundred twenty-nine of them were selected for long-term follow-up study by conducting random research on positive and negative sample sets. One hundred one patients with benign tumors and 42 patients with malignant tumors were found. In this paper, 42 samples were sampled for analysis. The final analysis results showed that there were 45 benign cases and 20 malignant cases after the test. In this paper, the collected information is classified and sorted, and the relevant characteristic results are obtained [8]. Then, the extracted training samples and verification samples are standardized, the label of malignant data is 0, and the label of benign is 1. Experimental data partitioning results are shown in Table 1.

RETRACTED

### 2.6. Feature Dimensionality Reduction and Modeling

In the whole process of the test, the eigenvalues in the dimension reduction step are correspondingly picked out in the model evaluation, and the data training is carried out according to the mainstream radionics method. It can be found that the calculated result in the threshold value is 0.865, which is accurate after calculation [9]. The rate reached 93%. Then, this paper uses the corresponding method for further analysis. When the threshold value is 0.93, it can be found that the feature vector has statistical significance in the regression model after analysis and calculation. The details are shown in Table 2.

### 2.7. Model Evaluation and Comparison

A vector machine trains the 32 image features selected in this paper with Gaussian kernel, and the butterfly model m0 and the ten features selected by LASSO are trained by mainstream methods. The model needs to have sufficient attribute induction ability and fitting ability to be brought into the three models. Figures 4 and 5 are the ROC curves of the three models in the training and validation sets. The curves in the figure show that the three models are relatively close in reclassification and prediction, and the difference is not significant.

## 3. Conclusion

Modeling verification experiments have proved that using the mainstream Spearman method to remove redundancy and dimensionality reduction sorting through SVM_RFE can effectively control erroneous diagnosis and treatment and excessive medical problems in the process of tumor diagnosis. Sex plays a perfect role in control.

## Figures and Tables

**Figure 1:** Framework of the overtreatment discovery diagnostic approach.

**Figure 2:** The training data extraction process based on similar expert prescriptions.

**Figure 3:** Digital imaging of lung nodules.

**Figure 4:** ROC curve on the training set.

**Figure 5:** ROC curve on the validation set.

**Table 1:** Experimental data partitioning results.

Label	Category 0	Category 1	Total/case
Training data	37	97	134
Verify the data	17	40	57

**Table 2:** Experimental results of three different dimensionality reduction and modeling methods on the training set.

Dimensionality reductionand modeling methods	Keep the numberof features	Accuracy (%)
LASSO + LR	10	83.70
Spearman + RFE + SVM	42	97.78
SVM_RFE + SVM	32	97.78

RETRACTED

## Data Availability

The data used to support the findings of this study are available from the corresponding author upon request.
